The article "Study on Various Luteal Characteristics Using Doppler Ultrasonography for Early Pregnancy Diagnosis in Nili-Ravi Buffaloes" was retracted in 2024. Reasons: signs of a paper mill; suspected computer-generated content; unreliable results or conclusions; concerns about the data.

# Study on Various Luteal Characteristics Using Doppler Ultrasonography for Early Pregnancy Diagnosis in Nili-Ravi Buffaloes

**DOI:** 10.1155/2022/3896068

**Published:** 2022-08-08

**Authors:** Umair Riaz, Mubbashar Hassan, Muhammad I. Khan, Umer Farooq, Farah Ali, Khalid Mehmood, Aftab Shaukat, Mushtaq H. Lashari, Liguo Yang

**Affiliations:** ^1^National Center for International Research on Animal Genetics, Breeding and Reproduction (NCIRAGBR), Huazhong Agricultural University, Wuhan, China; ^2^Department of Theriogenology, Faculty of Veterinary and Animal Sciences, The Islamia University of Bahawalpur, Punjab, Pakistan; ^3^Department of Clinical Sciences, University of Veterinary and Animal Science, Jhang Campus, Punjab, Pakistan; ^4^Department of Theriogenology, Faculty of Veterinary and Animal Sciences, University of Veterinary and Animal Sciences, Lahore, Punjab, Pakistan; ^5^Department of Physiology, Faculty of Veterinary and Animal Sciences, The Islamia University of Bahawalpur, Punjab, Pakistan; ^6^Department of Clinical Medicine and Surgery, Faculty of Veterinary and Animal Sciences, The Islamia University of Bahawalpur, Punjab, Pakistan; ^7^Department of Zoology, The Islamia University of Bahawalpur, Punjab, Pakistan

## Abstract

The objective of current study was to assess the trend in various luteal characteristics *viz* luteal size (LS), plasma progesterone (P^4^) concentration, and luteal blood flow (LBF) using color Doppler imaging (CDI) and power Doppler imaging (PDI) modes in pregnant and nonpregnant Nili-Ravi buffaloes. Lactating, cyclic, and healthy Nili-Ravi buffaloes (*n* = 09) without any reproductive abnormality were selected in present study. Buffaloes were synchronized using Ov-Synch, and fixed-time artificially insemination was performed (day = 0). Pregnancy was diagnosed on 30-day post-AI using B-mode ultrasonography based on presence or absence of embryonic heartbeat. Ovaries of all animals were scanned from day 5 till 21 post-AI using both B-mode and Doppler ultrasonography to measure LS and LBF. After each ovarian ultrasound examination, blood samples were collected via jugular venipuncture to determine plasma P^4^ concentration. According to results, LBF using CDI and PDI was significantly higher (*P* ≤ 0.05) in pregnant buffaloes on days 13 and 15 post-AI, respectively. The mean LS and plasma P^4^ concentration did not differ (*P* ≥ 0.05) between pregnant and nonpregnant animals until day 15 post-AI. However, a significant difference (*P* ≤ 0.05) was noticed for both on day 17 and onwards. It is concluded that LBF is a more sensitive luteal character as compared to LS and P^4^ for earlier pregnancy diagnosis in Nili-Ravi buffaloes when ascertained through CDI.

The article "Study on Various Luteal Characteristics Using Doppler Ultrasonography for Early Pregnancy Diagnosis in Nili-Ravi Buffaloes" was retracted in 2024. Reasons: signs of a paper mill; suspected computer-generated content; unreliable results or conclusions; concerns about the data.

## 1. Introduction

Despite having a significant share in world's milk supply (97,417,135 tons/annum) [1], buffalo dairy production is affected by its reproductive attributes such as delayed puberty, seasonal breeding pattern, less pronounced estrus, variable time of ovulation, high embryonic mortality, and increased calving interval [2, 3]. Milk yield per day is reduced significantly with the increase in calving interval resulting in economic losses [4]. In order to achieve economic viability and sustained milk production, a calving interval of ≤400 days should be attained [5]. Early detection of nonpregnant animals and their reinsemination of is a key to achieve the goal of one calf per year [6].

The most reliable mean of pregnancy diagnosis in buffaloes is transrectal B-mode ultrasonography conducted around 24 to 30 days post-breeding [7, 8]. Similarly, other chemical based methods have also been reported to detect pregnancy in buffaloes and rely on quantification of progesterone (P^4^) in milk and blood at around day 24 post-AI [9]. Pregnancy associated glycoproteins (PAGs) have also been reported for pregnancy diagnosis in buffalo with acceptable accuracy around day 25 postbreeding [10]. Apart from difficulty in conducting chemical-based methods under the field conditions, these methods require repeated sampling and are useful only after maternal recognition of pregnancy that takes place at around day 17 postbreeding [11].

Corpus luteum (CL) has a highest blood supply per tissue volume compared to all other organs, and angiogenesis increases with the growth of CL. In comparison to B-mode, color Doppler ultrasonography is a reliable method to monitor the information related to blood flow of an organ or tissue [12]. Color Doppler ultrasonography has widened the scale of diagnostic imaging from structural to functional aspect in bovine [13]. Modern color Doppler ultrasound scanners are equipped with two techniques *viz* color Doppler imaging (CDI) and power Doppler imaging (PDI) to analyze the blood flow where the latter is considered more sensitive and freer of aliasing artifacts. Hence, PDI is considered advantageous for measuring luteal blood flow (LBF) in cows [14], however, no such information is yet available in Nili-Ravi buffaloes.

Color Doppler ultrasonography has emerged as useful technique to quantify LBF for early identification of nonpregnant animals and for their subsequent reinseminations. Several studies in *Bos taurus* [15], *Bos indicus* [16], and in Mediterranean and Egyptian buffaloes have suggested that LBF is as an indicator of early pregnancy diagnosis [17, 18]; however, these studies on buffaloes lack in depth analysis of LBF and involve postbreeding monitoring of CL for a short or limited time-period with few observations. Moreover, comparative information on luteal dynamics of pregnant and nonpregnant Nili-Ravi buffaloes is not available to date. The objective of current study was to assess the trend in various luteal characteristics *viz* luteal size (LS), plasma progesterone (P^4^) concentration, and luteal blood flow (LBF) using color Doppler imaging (CDI) and power Doppler imaging (PDI) modes in pregnant and nonpregnant Nili-Ravi buffaloes.

The article "Study on Various Luteal Characteristics Using Doppler Ultrasonography for Early Pregnancy Diagnosis in Nili-Ravi Buffaloes" was retracted in 2024. Reasons: signs of a paper mill; suspected computer-generated content; unreliable results or conclusions; concerns about the data.

## 2. Materials and Methods

### 2.1. Compliance with Ethical Standards

Current study was performed in accordance with regulations provided by Animal Ethics Board of Huazhong Agricultural University; Grant no. (HZAUMO_2015-12), Wuhan, China. The experimental design was carried out according to good veterinary practices under farm conditions. Besides this, all possible care of animals was taken to ensure maximum welfare.

### 2.2. Animal Care and Management

Present study was carried out during the breeding season (September to December 2020) at Buffalo Research Institute, Pattoki, District Kasur, Punjab, Pakistan. Clinically healthy Nili-Ravi buffaloes (*n* = 09) of mixed-parity, with a mean (±SE) body weight of 432.5 ± 23.4 kg, lactating, and having mean (±SE) postpartum days of 163.2 ± 16.2 were selected. All buffaloes were having a regular estrous cycle and had no palpable abnormality in their reproductive tract. Mean body condition score (BCS) of buffaloes was 3.5 ± 0.4 on a 1–5 point scale (5-point scale: 1 = emaciated and 5 = obese) [19]. The buffaloes were kept under semicovered housing with free access to water, offered 30–40 kg of green fodder, 1-2 kg of concentrate comprising of 15% crude protein, and 65% total digestible nutrients per buffalo on daily basis.

### 2.3. Estrus Synchronization Protocol

All buffaloes were synchronized using Ov-Synch protocol in which 1^st^ GnRH injection (lecirelin 50 *μ*g/2 cc, I/M. Dalmarelin™ Fatro Co., Italy) was administered to buffaloes at a random day of estrous cycle followed by PGF_2_*α* injection (cloprostenol 150 *μ*g/2 cc, I/M. Dalmazin™ Fatro Co. Italy) at an interval of 7 days. A second injection of GnRH was administered 48 h after PGF_2_*α*, and fixed-time artificial insemination (AI) was performed after 16 h of the last GnRH injection and considered as day 0 in this study [20].

### 2.4. Ovarian B-Mode and Doppler Sonography for Luteal Dynamics

All buffaloes were subjected to ovarian ultrasound with B-mode and color Doppler mode scanning (My Lab™ 30 VET Gold, Esaote, Genoa, Italy) on alternated days from day 5 to 21 post-AI by a same operator to measure the LS and blood flow pattern. Initially, a linear array transducer (7.5 MHz) was used to scan LS using B-mode ultrasound; later, LBF was measured in the same cross-sectional image of CL by activating Doppler mode ultrasound. Each cross section was examined with both color (CDI) and power (PDI) modes of Doppler ultrasound (see Figure 1). For each animal, three separate observations were recorded using B-mode, CDI, and PDI. All images were stored in bitmap-format in ultrasound machine and transferred to universal storage drive. Thus, each buffalo was scanned 9 times, resulting in a total of 81 measurements. Buffaloes were retrospectively classified as pregnant (presence of embryonic heartbeat, *n* = 4) or nonpregnant (absence of embryo, *n* = 5) on day 30 after AI with B-mode ultrasound.

The article "Study on Various Luteal Characteristics Using Doppler Ultrasonography for Early Pregnancy Diagnosis in Nili-Ravi Buffaloes" was retracted in 2024. Reasons: signs of a paper mill; suspected computer-generated content; unreliable results or conclusions; concerns about the data.

### 2.5. Image Analysis and Quantification

The stored images were examined using offline software “Image J” (National Health Institute, Bethesda, MD, USA). Diameter of CL was determined using B-mode images, as explained previously [21]. To measure the cross-sectional area, CL was cropped using “Image J” for pixel analysis. Similarly, using the same software, the area of color pixels within the CL was quantified, which was considered as a semiquantitative parameter of LBF. In each examination, mean values of three images were taken to minimize the chance of error.

### 2.6. Blood Samples and Progesterone Assay

After each ovarian ultrasound examination, blood samples were collected via jugular venipuncture in vacutainer tubes containing heparin (Vacutainer ® Systems Europe, Becton Dickinson, Meylan Cedex, France). Centrifugation of blood samples was performed at 4100 g for 10 mins, and the plasma was stored at −80°C until further analysis. Plasma concentrations of P^4^ were measured by using a commercially available double antibody radioimmunoassay kit (Immunotech, Prague, Czech Republic) with a 125I-labelled tracer. The interassay and intraassay coefficients of variation for P^4^ assay were 6.2% and 3.5%, respectively, with a minimum detection limit of 0.3 ng/ml.

### 2.7. Statistical Analysis

Normal distribution of the data was verified using Kolmogorov-Smirnov and Shapiro-Wilk tests. Data is presented as mean (± SE). The difference between different days and between pregnant and nonpregnant groups for LS, P^4^ and LBF was ascertained through analysis of variance (ANOVA) of repeated measure followed by least significant difference (LSD) as a post hoc test. Probability level of *P* ≤ 0.05 was considered significant. Relationship between and among various studied attributes was deduced using Pearson's correlation coefficient, and accordingly, the regression equations were derived through regression analyses. All data were analyzed using Statistical Package for Social Sciences (SPSS for Windows Version12, SPSS Inc., Chicago, IL, USA).

The article "Study on Various Luteal Characteristics Using Doppler Ultrasonography for Early Pregnancy Diagnosis in Nili-Ravi Buffaloes" was retracted in 2024. Reasons: signs of a paper mill; suspected computer-generated content; unreliable results or conclusions; concerns about the data.

## 3. Results

Changes in LS, LBF (CDI, PDI), and P^4^ during day 5 to 21 postinsemination in nonpregnant Nili-Ravi buffaloes are presented in Table 1. The mean (±SE) LS increased nonsignificantly (*P* ≥ 0.05) till day 9 post-AI and began to increase significantly (*P* ≤ 0.05) from day 11 till 17 post-AI in nonpregnant buffaloes. Afterward, CL size was found to be decreased (*P* ≤ 0.05) on day 19 post-AI. The mean (±SE) plasma P^4^ concentration and LBF (both with CDI and PDI) increased significantly (*P* ≤ 0.05) from day 9 and 11, respectively, till day 17 post-AI, after which a decrease (*P* ≤ 0.05) in P^4^ concentration and LBF was observed on day 19 post-AI in nonpregnant Nili-Ravi buffaloes.

Changes in LS, LBF (CDI, PDI), and P^4^ during day 5 to 21 postinsemination in pregnant Nili-Ravi buffaloes are presented in Table 2. The mean (±SE) LS increased significantly (*P* ≤ 0.05) on day 7 to 21 post-AI. The mean CDI increased significantly (*P* ≤ 0.05) from day 7 post-AI, while significant increase in mean PDI and plasma P^4^ concentrations was observed from day 9 to 21 post-AI in pregnant buffaloes.

A comparison between LS, LBF (CDI, PDI), and P^4^ between pregnant and nonpregnant Nili-Ravi buffaloes is presented in Figure 2. The mean (± SEM) LS and plasma P^4^ concentration did not differ between pregnant and nonpregnant animals until day 15 post-AI. However, a significant difference was noticed on day 17 (*P* ≤ 0.05) onwards (see Figures 2(a) and 2(b)). The mean LBF with CDI and PDI significantly differed (*P* ≤ 0.05) at day 13 and 15 post-AI between pregnant and nonpregnant buffaloes, respectively (see Figures 2(c) and 2(d)).

Correlation coefficients between LS, CDI, PDI, and P^4^ in pregnant and nonpregnant Nili-Ravi buffaloes are presented below (see Table 3). All CL attributes were positively correlated to each other, and highest values were found for CDI × PDI in nonpregnant buffaloes (*r* = 0.7030, adjusted *R*^2^ = 0.48, *P* ≤ 0.01) and for CDI × PDI and CDI × P^4^ in pregnant buffaloes (*r* = 0.98, adjusted *R*^2^ = 0.97, *P* ≤ 0.01).

## 4. Discussion

The current study reports the relative changes between LS, plasma P^4^ concentration, and LBF measured with two methods (CDI and PDI) in pregnant and nonpregnant Nili-Ravi buffaloes over the period of CL development and regression after insemination. Previously, fewer studies with different timeframes of CL measurements have been reported in Italian and Egyptian buffaloes [18, 22]. However, assessment of CL attributes using Doppler imaging during its growth and regression phases has not yet been reported for pregnant and nonpregnant Nili-Ravi buffaloes.

The article "Study on Various Luteal Characteristics Using Doppler Ultrasonography for Early Pregnancy Diagnosis in Nili-Ravi Buffaloes" was retracted in 2024. Reasons: signs of a paper mill; suspected computer-generated content; unreliable results or conclusions; concerns about the data.

The key finding of the present study is that LBF, either measured with CDI or PDI, is a better indicator of luteal function and early pregnancy as compared to LS or plasma P^4^ concentration between pregnant or nonpregnant Nili-Ravi buffaloes. The reason is that LBF begins to differ relatively earlier with CDI on day 13 and with PDI on day 15 post-AI, whereas the LS and plasma P^4^ concentration showed divergence on day 17 post-AI between pregnant and nonpregnant Nili-Ravi buffaloes. This is in accordance with earlier report for Egyptian buffaloes and dairy cows in which a significantly higher LBF after AI was observed on day 14 and 15, respectively, and was associated with pregnancy [18, 23]. Studies on *Bos taurus and Bos indicus* have also reported similar changes in LBF of pregnant animals as compared to nonpregnant ones [15, 16]. Higher level of LBF in pregnant animals could be attributed to increased vascularity of luteal tissue owing to elevated demand of P^4^ concentration for embryonic support during the pregnancy [24].

In the current study, all functional traits of CL were observed to maintain an increasing trend in pregnant Nili-Ravi buffaloes during the critical period of maternal recognition of pregnancy which takes place around day 15-18 after AI [25]. On the other hand, buffaloes that failed to maintain pregnancy exhibited a decline in CL attributes around day 17 post-AI. This is in accordance with previous studies conducted in beef heifers and dairy cows emphasizing that newly flourishing embryo releases interferon tau (IFNT) before its attachment to uterine wall which in turns blocks the release of PGF2*α* from uterine endometrium to prevent luteolysis [11, 26, 27]. During the critical time of maternal recognition of pregnancy, an increased LBF facilitates the relay of embryonic message to prevent luteolysis. This maintains the luteal function of P^4^ production at the time of maternal recognition of pregnancy through the utero-ovarian circulation [11].

In the present study, significant increase in LS took place quite earlier (day 7 post-AI) in pregnant buffaloes as compared to that of nonpregnant ones whereas LS remained consistent till day 11 post-AI. Earlier reports in Mediterranean buffaloes have also concluded that CL dimensions in pregnant buffaloes increased between day 5 to 10 post-AI, and it can be used to predict the early established pregnancy compared to absolute size of CL [17, 22]. It has been reported that CLs which exhibit early development have greater expression of endothelial growth factor resulting in an increased angiogenesis and increased LBF [22].

The article "Study on Various Luteal Characteristics Using Doppler Ultrasonography for Early Pregnancy Diagnosis in Nili-Ravi Buffaloes" was retracted in 2024. Reasons: signs of a paper mill; suspected computer-generated content; unreliable results or conclusions; concerns about the data.

Results of the current study indicate that the LBF either measured with CDI or PDI turns out to be a good indicator of luteal function as compared to LS and plasma P^4^ concentration. This could be due to steady growth in luteal vasculature of pregnant buffaloes which has been reported to increase up to 25% between day 6 and 12 postovulation in bovine ovary [28]. In the current study, LBF values with CDI and PDI did not differ significantly on any specific day of observation. Similar observation about PDI have been reported, and it has been suggested that PDI is more sensitive for LBF measurements. This variation could be due to limited number of sample size in the present study [14].

In the current study, functional traits of CL exhibited strong correlation among each other. The obvious reason of strong interrelationship among the attributes studied is that all these parameters are dependent on the functionality of one glandular organ which is CL. These findings are in agreement with previous studies in dairy cows and heifers reporting high correlation among CL attributes [15, 16, 27].

## 5. Conclusions

It is concluded that color Doppler ultrasonography of CL postbreeding can be utilized to predict early pregnancy in Nili-Ravi buffaloes. Among functional traits of CL, the LBF tends to be more sensitive and diverges earlier than LS and plasma P^4^ concentration between pregnant and nonpregnant Nili-Ravi buffaloes. These findings could be implied to rebreed buffaloes that fail to become pregnant without wasting successive estrus. In this way, these findings would be helpful in reducing calving interval and increase reproductive efficiency for an economically sustainable buffalo farming.

## Figures and Tables

**Figure 1:** Representative ultrasound images of corpus luteum (CL) in Nili-Ravi buffaloes on day 5 postinsemination. (a) B-mode ultrasound image of CL taken by 7.5 MHz transrectal transducer. (b) Color Doppler image depicting luteal blood flow of day 5 postinsemination CL. (c) Power Doppler image depicting luteal blood flow of Day 5 post-insemination CL. The white dotted circles indicate the area of interest (AOI) used to calculate the cross-sectional area of the CL. Within the AOI, the coloured pixels were quantified using image J software (National Institute of Health, Bethesda, MD, USA) to assess the luteal blood flow.

**Figure 2:** Comparison of various CL parameters between pregnant and nonpregnant Nili-Ravi buffaloes after artificial insemination (day 0) from days 5 to 21. (a) Luteal size. (b) Plasma progesterone concentration. (c) Luteal blood flow measured with Color Doppler Imaging (CDI). (D) Luteal blood flow measured with power Doppler imaging (PDI). Different letters (a, b) indicate significant (*P* ≤ 0.05) differences between the groups.

The article "Study on Various Luteal Characteristics Using Doppler Ultrasonography for Early Pregnancy Diagnosis in Nili-Ravi Buffaloes" was retracted in 2024. Reasons: signs of a paper mill; suspected computer-generated content; unreliable results or conclusions; concerns about the data.

**Table 1:** Comparison of luteal size (LS), plasma progesterone (P^4^) concentration, and luteal blood flow (LBF) monitored with color and power Doppler imaging (CDI and PDI) in nonpregnant Nili-Ravi buffaloes (*n* = 5) from day 5 to 21 post-AI.

Days	LS (cm^2^)	P^4^ (ng/ml)	LBF	
			CDI (cm^2^)	PDI (cm^2^)
5	1.4 ± 0.1^a^	1.8 ± 0.3^a^	0.4 ± 0.07^a^	0.4 ± 0.06^a^
7	1.6 ± 0.1^a^	2.8 ± 0.4^a^	0.6 ± 0.08^a^	0.6 ± 0.06^a^
9	1.9 ± 0.07^a^	3.5 ± 0.4^b^	0.6 ± 0.05^a^	0.7 ± 0.4^a^
11	2.1 ± 0.09^b^	4.4 ± 0.6^b^	0.8 ± 0.08^b^	0.9 ± 0.1^b^
13	2.5 ± 0.1^b^	5.3 ± 0.6^b^	1.0 ± 0.1^b^	1.0 ± 0.1^b^
15	2.4 ± 0.1^b^	4.8 ± 0.6^b^	0.9 ± 0.1^b^	0.9 ± 0.1^b^
17	1.9 ± 0.1^b^	4.0 ± 0.6^b^	0.8 ± 0.1^b^	0.8 ± 0.09^b^
19	1.6 ± 0.2^a^	2.7 ± 0.6^a^	0.5 ± 0.05^a^	0.5 ± 0.02^a^
21	1.2 ± 0.2^a^	1.0 ± 0.4^a^	0.2 ± 0.01^a^	0.3 ± 0.03^a^

Values are expressed as mean ± standard error. ^a,b^ in rows indicate differences (*P* < 0.05) between CL parameters for a given day post-AI.

**Table 2:** Comparison of luteal size (LS), plasma progesterone (P^4^) concentration, and luteal blood flow (LBF) monitored with color and power Doppler imaging (CDI and PDI) in pregnant Nili-Ravi buffaloes (*n* = 4) from day 5 to 21 post-AI.

Days	LS (cm^2^)	P^4^ (ng/ml)	LBF	
			CDI (cm^2^)	PDI (cm^2^)
5	1.3 ± 0.2^a^	1.6 ± 0.2^a^	0.5 ± 0.05^a^	0.5 ± 0.07^a^
7	1.8 ± 0.1^b^	2.3 ± 0.3^a^	0.7 ± 0.03^b^	0.8 ± 0.1^a^
9	2.1 ± 0.1^b^	4.1 ± 0.6^b^	0.8 ± 0.1^b^	0.9 ± 0.08^b^
11	2.6 ± 0.2^b^	4.6 ± 0.4^b^	1.1 ± 0.1^b^	1.1 ± 0.1^b^
13	2.7 ± 0.1^b^	5.7 ± 0.7^b^	1.±0.06^b^	1.4 ± 0.1^b^
15	2.7 ± 0.1^b^	6.1 ± 0.7^b^	1.5 ± 0.06^b^	1.5 ± 0.1^b^
17	2.8 ± 0.1^b^	6.2 ± 0.5^b^	1.6 ± 0.01^b^	1.7 ± 0.1^b^
19	2.9 ± 0.1^b^	6.4 ± 0.7^b^	1.8 ± 0.06^b^	1.9 ± 0.1^b^
21	3.2 ± 0.1^b^	6.9 ± 0.5^b^	2.1 ± 0.06^b^	2.0 ± 0.1^b^

Values are expressed as mean ± standard error. ^a,b^ in rows indicate differences (*P* < 0.05) between CL parameters for a given day post-AI.

**Table 3:** Correlations coefficients among various CL parameters (LS, P^4^, PDI, and CDI) in pregnant and nonpregnant Nili-Ravi buffaloes.

CL parameters	*r* value	Adjusted *R*^2^	Regression equation
Nonpregnant (*n* = 5)			
LS × CDI	0.545^∗∗^	0.28	*Y* = 0.8 *x* + 1.2
LS × PDI	0.610^∗∗^	0.35	*Y* = 1.08*x* + 1.1
LS × P^4^	0.554^∗∗^	0.29	*Y* = 1.7*x* + 1.2
CDI × PDI	0.703^∗∗^	0.48	*Y* = 0.7*x* + 0.1
CDI × P^4^	0.567^∗∗^	0.30	*Y* = 0.1*x* + 0.3
PDI × P^4^	0.390^∗∗^	0.13	*Y* = 0.06*x* + 0.4
Pregnant (*n* = 4)			
LS × CDI	0.804^∗∗^	0.63	*Y* = 0.9*x* + 1.2
LS × PDI	0.735^∗∗^	0.52	*Y* = 0.8*x* + 1.4
LS × P^4^	0.755^∗∗^	0.55	*Y* = 0.2*x* + 1.4
CDI × PDI	0.988^∗∗^	0.97	*Y* = 0.9*x* − 0.2
CDI × P^4^	0.988^∗∗^	0.97	*Y* = 0.9*x* − 0.2
PDI × P^4^	0.961^∗∗^	0.91	*Y* = 0.2*x* − 0.1

^∗∗^Correlation is significant at *P* ≤ 0.01. LS: luteal size; PDI: power Doppler imaging; CDI: color Doppler imaging; P^4^: progesterone.

The article "Study on Various Luteal Characteristics Using Doppler Ultrasonography for Early Pregnancy Diagnosis in Nili-Ravi Buffaloes" was retracted in 2024. Reasons: signs of a paper mill; suspected computer-generated content; unreliable results or conclusions; concerns about the data.

## Data Availability

The numerical data used to support the findings of this study are available from the corresponding author upon request.
